RETRACTED

# Application Value of the CT Scan 3D Reconstruction Technique in Maxillofacial Fracture Patients

**DOI:** 10.1155/2022/1643434

**Published:** 2022-07-07

**Authors:** Jie Kang, Lijie Jiang

**Affiliations:** Department of Image Center, Hengshui People's Hospital, Hengshui, Hebei, China

## Abstract

*Purpose* The aim of the study was to explore the application value of computerized tomography (CT) scan 3D reconstruction technology in maxillofacial fracture patients. *Methods* A total of 80 maxillofacial fracture patients who underwent surgical treatment in Shijiazhuang People's Hospital from January 2019 to January 2020 were enrolled. All of them received 128-slice spiral CT  scans before surgery, and the images were subjected to multiplanar reconstruction (MRP) and volume reconstruction (VR). *Results* A total of 181 fractures were found in 80 patients with maxillofacial fractures. The detection rates of axial CT, MRP, and VR were 77.90% (141/181), 93.92% (170/181), and 97.79% (177/181), respectively. The detection rates of the four inspection methods were statistically different. Taking the findings of surgical anatomy as the gold standard, the sensitivity of MRP and VR for the diagnosis of maxillofacial fractures was 90.06% (163/170) and 95.56% (174/177), with no significant difference. *Conclusion* CT scan 3D reconstruction technology has a high application value in the clinical diagnosis and treatment of maxillofacial fracture patients.

## 1. Introduction

Maxillofacial region is prone to fracture after trauma, and a comprehensive understanding of the fracture is therefore of great significance to formulate an appropriate surgical schedule [1]. The complicated anatomical structure of the maxillofacial region challenges and obscures correct judgment of the fracture type [2,3]. Due to the anatomical relationship of maxillofacial bone and the displacement of fracture, the resolution and accuracy of ordinary X-ray films are poor and show compound overlapping images of multiple structures [4]. Multislice spiral CT (MSCT) is a noninvasive imaging examination technology, and it can display human bones, joints, soft tissues, blood vessels, and other aspects more clearly and effectively prevent the image clarity of motion artifacts owing to its high scanning speed in unit time [5,6]. However, for the complex layer of the maxillofacial region, it is difficult for an ordinary MSCT scan to perform specific display. Therefore, it needs to use the postprocessing technology of the MSCT scan to perform intuitive and three-dimensional display [7,8]. There are various imaging methods of MSCT postprocessing, among which multiplanar reconstruction (MRP) and volume reconstruction (VR) are more well recognized [9]. With the optimization of related technologies in recent years, CT scan 3D reconstruction has gradually become the trend in the diagnosis and treatment of the maxillofacial fracture [10]. CT scan 3D reconstruction technology can fully display the fractured status, allowing the doctor to observe from multiple angles and all directions, and thus providing a scientific basis for the subsequent surgical plan [11,12]. Accordingly, in the present study, we aimed to explore the significance of CT scan 3D reconstruction for the diagnosis of maxillofacial fractures.

RETRACTED

## 2. Materials and Methods

### 2.1. Study Population

A total of 80 maxillofacial fracture patients who underwent surgical treatment in our hospital from January 2019 to January 2020 were selected, including 45 males and 35 females, aged 28–65 years old, with an average age of (39.23 ± 7.21) years old. The cause of injury included 32 cases of traffic accidents, 24 cases of fall injuries, 17 cases of beating injuries, and 7 cases of other causes. The study was approved by the Ethics Committee of Shijiazhuang People's Hospital, (approved no. sjz7331), and the patients signed an informed consent form.

### 2.2. Inclusion and Exclusion Criteria

#### 2.2.1. Inclusion Criteria

The inclusion criteria were as follows: (a)those who met the clinical diagnostic criteria of the maxillofacial fracture; (b) the fracture types were Le Fort I∼III [13]; (c) 64-slice spiral CT examination was performed before operation.

#### 2.2.2. Exclusion Criteria

The exclusion criteria were as follows: (a) patients with pathological or old fracture; (b) patients with neurological disease or cognitive dysfunction; (c) patients with poor compliance with the research; (d) patients with contraindications for CT examination.

### 2.3. Method

The patient took the supine position, and the Brilliance 128-slice spiral CT scanner produced by Philips in the Netherlands was used to scan the lateral position of the head. The scanning range was 4 cm from the upper orbital edge to 4 cm from the lower edge of the mandible. Parameter setting is as follows: tube voltage 120 kV, tube current 220 mA, and duration 3∼4s; after scanning, the original data were reconstructed, the layer thickness was 0.5 mm, the layer spacing was 0.3 mm, and the matrix was 512 × 512. The reconstructed data were transmitted to the instrument workstation for three-dimensional postprocessing, and the images were subjected to MRP and VR. MRP was to superimpose all the axial images in the scanning range and then reorganize some markings of the tissue designated by the line reorganized in coronal, sagittal, and oblique images at any angle. VR was to make the assumed projection line pass through the scanning volume at a given angle and comprehensively display the pixel information in the volume. All images were evaluated by 3 radiologists with more than 4 years of clinical experience, using a double-blind method. In case of disagreement, the decision shall be made by voting to obtain the diagnosis conclusion.

RETRACTED

### 2.4. Observation Indicators

Based on the surgical results, the number of fracture sites was calculated. Fracture sites included maxillary fracture, mandibular fracture, zygomatic fracture, orbital fracture, nasal bone fracture, sphenoid fracture, and temporomandibular joint dislocation. The number of different fracture types and the detectable rate of axial CT, MPR, and VR were calculated.

### 2.5. Statistical Methods

The data were processed by the SPSS22.0 statistical software, and the graphics were plotted by GraphPad prism 8.0. The count data were expressed as (%) and analysed by the *χ*2 test. *P* < 0.05 suggested a statistically significant difference.

## 3. Results

### 3.1. Results of Maxillofacial Fractures

A total of 181 fractures were found in 80 patients with maxillofacial fractures, including 43 maxillary fractures, 28 mandibular fractures, 43 zygomatic fractures, 28 orbital fractures, 34 nasal fractures, 3 sphenoid fractures, and 2 dislocations of the temporomandibular joint (Table 1).

### 3.2. Detection Rate of MRP and VR

A total of 141 sites were detected in axial CT, 170 sites were detected in MRP, and 177 sites were detected in VR. The detection rates of MRP and VR were higher than that of the axial CT, and the detection rate between MRP and VR had no difference (Table 2).

### 3.3. Diagnosis Sensitivity of MRP and VR

In MRP, 163 sites were confirmed by surgery with 7 sites being false positive, while 173 sites in VR were confirmed by surgery with 4 sites being false positive. There was no significant difference in diagnosis sensitivity between the two groups (*P* > 0.05) (see Table 3).

## 4. Discussion

Maxillofacial fractures cause facial dysfunction of patients and adversely impact their appearance. Therefore, an appropriate treatment plan to improve the prognosis is of an urgent need. Due to the complex structure of the maxillofacial region, the conventional examination cannot clearly and comprehensively show the fracture. As a result, it requires a thorough understanding of the spatial relationship of the maxillofacial fractures to carry out the treatment plan. Traditional examination methods, such as X-ray, are insufficient to reduce the incidence of clinical misdiagnosis. The results of this study showed that the detection rate of maxillofacial fractures by axial CT was 77.90%, of which the detection rate of zygomatic fractures (83.72%) was the highest, followed by nasal bone fractures (82.35%), and the detection rate of temporomandibular joint dislocations was lower. It might be due to the limitation of axial CT in showing the relationship between the three-dimensional structure of the fracture and the surrounding tissues. Thus, more precise and efficient inspection methods are highly desired to enhance the diagnosis and the treatment effect.

RETRACTED

With the optimization of medical technology, CT scan 3D reconstruction technology is gradually popularized in the diagnosis and treatment of maxillofacial fractures [14]. With the powerful postprocessing capabilities, it can rebuild the maxillofacial fracture, enable the doctor to understand the fracture location, fracture line direction, and fracture displacement [15]. Thus, it provides a more scientific imaging basis for the treatment plans. MPR, one of the CT scan 3D reconstruction techniques, could clearly show the fracture position, yet with poor 3D perception. In this study, the detection rate of maxillofacial fractures by MRP was 93.92%, among which sphenoid fractures (100.00%) and temporomandibular joint dislocations (100.00%) had the highest detection rates, followed by zygomatic fractures (97.67%), nasal bones fractures (94.12%), mandibular fractures (92.86%), orbital fractures (92.86%), and maxillary fractures (90.70%). The finding can be attributed to the fact that MRP reconstructs the fracture position from any angle such as sagittal, coronal, oblique, and curved planes [16]. In addition to MPR, VR is one of the most eye-catching emerging technologies in recent years [17]. In this study, the detection rate of VR on maxillofacial fractures was 97.79%, and the rate was the highest in mandibular fractures (100.00%), zygomatic fractures (100.00%), orbital fractures (100.00%), sphenoid fractures (100.00%), and dislocations of the temporomandibular joint (100.00%). Compared with MRP, it increases the detection rate of mandibular fractures, zygomatic fractures, and orbital fractures. Possibly, it can compensate for the deficiency of MPR, the three-dimensional display of the anatomical structure, and fracture images of the maxillofacial region and thus providing a more intuitive and three-dimensional understanding of the relationship between the broken end and the spatial structure of the surrounding tissues [18,19]. Similarly, Alessa concluded that the detection rate of MPR plus VR was superior to that of axial CT (99.5% (209/210) vs 88.1% (185/210)), confirming that CT scan 3D reconstruction technology has a reliable value [20]. In addition, with the results of surgical anatomy as the gold standard, the sensitivity of MRP and VR for the diagnosis of maxillofacial fractures was 90.06% (163/170) and 95.56% (174/177), respectively, with no significant difference.

RETRACTED

## 5. Conclusion

CT scan 3D reconstruction is a reliable technique in the clinical diagnosis of maxillofacial fracture patients.

## Figures and Tables

**Table 1:** Results of maxillofacial fractures

Fracture site	Surgery	Axial CT	MRP	VR
Maxillary fractures	43	33	39	42
Mandibular fractures	28	19	26	28
Zygomatic fractures	43	36	42	43
Orbital fractures	28	22	26	28
Nasal bone fracture	34	28	32	31
Sphenoid fracture	3	2	3	3
Temporomandibular joint dislocation	2	1	2	2
Total	181	141	170	177

**Table 2:** Detection rate of MRP and VR.

	Total	Detected	Undetected	Detection rate
Axial CT	181	141	40	77.90%
MRP	181	170	11	93.92%^*∗*^
VR	181	177	4	97.79%^*∗*^
*χ*2				44.22
*P*				<0.001

*Note.* Compared with axial CT, the difference was statistically significant (*P* < 0.05).

**Table 3:** Diagnosis sensitivity of MRP and VR.

	Surgery		Sensitivity (%)
	+	-	
MRP (*n* = 170)	163	7	90.06%
VR (*n* = 177)	173	4	95.56%
*χ*2			0.975
P			0.323

## Data Availability

The datasets used and analysed during the current study are available from the corresponding author on reasonable request.
